This article has been retracted.

# Employing of Curcumin–Silver Nanoparticle-Incorporated Sodium Alginate-Co-Acacia Gum Film Hydrogels for Wound Dressing

**DOI:** 10.3390/gels9100780

**Published:** 2023-09-25

**Authors:** Fahad M. Aldakheel, Dalia Mohsen, Marwa M. El Sayed, Mohammed H. Fagir, Dalia K. El Dein

**Affiliations:** 1 Department of Clinical Laboratory Sciences, College of Applied Medical Sciences, King Saud University, Riyadh 11433, Saudi Arabia; faldakheel@ksu.edu.sa; 2 Clinical Laboratory Sciences Program, Inaya Medical College, Riyadh 12211, Saudi Arabia; husseinfagir@inaya.edu.sa (M.H.F.); dkmohammed@inaya.edu.sa (D.K.E.D.); 3 Microbiology Department, National Research Centre, Giza 12622, Egypt; 4 Chemical Engineering and Pilot Plant Department, National Research Centre, Giza 12622, Egypt; dr.marwameid@gmail.com

**Keywords:** chronic wounds, curcumin, silver, silver nanoparticles, Arabic gum hydrogel

## Abstract

Skin wound healing is time-consuming and frequently accompanied by bacterial infections and the development of scars. The rise of antibiotic-resistant bacterial strains has sparked a growing interest in naturally occurring bioactive substances, like curcumin, that possess wound-healing capabilities. Silver is a natural antimicrobial agent, and finds extensive use in specialized wound dressings. Silver nanoparticles (AgNPs) were synthesized using an eco-friendly approach, employing curcumin. The prepared nanoparticles have been characterized using TEM, DLS, and zeta potential. The prepared AgNPs were loaded on sodium alginate-co-gum arabic hydrogel. Two hydrogel samples (with and without AgNPs) have been applied for wound healing. The developed silver nanoparticles that were created exhibited effective action against both types of bacteria, namely *Gram-negative* and *Gram-positive*. Alg-co-AG-AgNPs demonstrated faster wound healing rates compared to using the control hydrogel sample. The novel dressings of curcumin–silver nanoparticle-incorporated sodium alginate-co-gum arabic hydrogels (Alg-co-AG-AgNPs) exhibited exceptional biocompatibility and have the potential to serve as a wound dressing that possesses antibacterial properties and reduces scarring.

## 1. Introduction

Skin is the largest organ in the human body, as 10% of the total body weight is skin, and it serves as a barrier from the elements [1]. In addition to its function as a physical barrier, it also acts as a thermoregulator, fluid homeostat, sensory detector, and immunological watchdog. Generally, a complicated and dynamic process allows the human body to repair damaged skin with little scarring [2]. Coagulation and hemostasis, inflammation, proliferation, and remodeling are the four time-dependent phases that make up the different processes of acute tissue healing. But a variety of factors, including local ones (such as oxygenation, wound infection, foreign bodies, venous sufficiency, wound area, depth, and local tension and pressure) and systemic ones (for example, age and gender, ischemia, obesity, diseases, alcoholism, medications, stress, smoking, immunocompromised conditions, and nutrition), could prevent the healing process from progressing. Medical attention is required since a number of variables have an impact on wound healing [3].

Rapid bacteria elimination and broad-spectrum antibacterial properties are essential for wound dressings in order to prevent and treat wound infection. The skin barrier is compromised in a wound, just like it is in the early stages of hemostasis, and the clotting blood acts as a fertile environment for the growth of invasive germs. A fresh wound, therefore, naturally has a significant risk of bacterial invasion and contamination. Numerous antibacterial substances, including medicines and silver ions, have been applied to wounds as bactericidal substances. However, their overall effectiveness in avoiding wound infection still does not meet therapeutic standards because of their constrained bactericidal range or the relatively sluggish bactericidal activity. Antibacterial peptides (AMPs) have been thoroughly investigated as possible antibacterial agents against common Gram-positive and Gram-negative bacteria, fungi, and protozoa, revealing broad-spectrum antimicrobial activity with favorable effectiveness [4,5].

Natural polymers (hydrogel) exhibit advantages in terms of biocompatibility and cost-effectiveness [6]. Hydrogels are synthesized using different types of polymers. Sodium alginate is one of the polymers which has been used for hydrogel preparation. Sodium Alginate is a prevalent natural polymer used in hydrogels, characterized by linear polysaccharide chains containing segments of (1,4)-linked β-D-mannuronic acid (M) and α-L-guluronic acid (G) residues. These G-blocks form intermolecular cross-links with divalent cations like Ca^2+^ to establish hydrogel structures [7]. Alginate-based hydrogels release small molecules and proteins, and offer bioactive ligands to cells. This type of hydrogel is degraded at controllable rates. Nonetheless, their stretchability is limited (they rupture when stretched to around 1.2 times their original length), rendering them somewhat brittle. The authors of [8] introduced a stretchable and robust hydrogel by combining ionically cross-linked alginate with covalently cross-linked polyacrylamide. Furthermore, the integration of nanoparticles into hydrogels has been explored to enhance adhesion and mechanical properties [9]. Acacia gum (also known as Arabic gum) is a natural biopolymer, possessing intricate and branched polymeric configurations that grant it significant adhesive characteristics. These attributes have led to extensive applications of gum in the food industry, where it serves as a dietary fiber [10], as well as in pharmaceutical constructions, fulfilling roles as a suspending agent, emulsifying agent, and contributing to its presence in cosmetics as a demulcent and emollient.

The “material of the 21st century” is thought to be nanoparticles (NPs), which have been studied for a variety of biomedical applications in recent decades and are regarded as such because of their distinctive designs and property combinations in comparison to traditional materials [11]. NPs have a wide range of uses, including in environmental research, engineering, electronics, medical applications, industrial domains, and human health appliances. In general, using nanoparticles as drug delivery systems has many advantages over using other drug delivery systems. Silver nanoparticles (AgNPs) are the most often employed form of metallic NPs due to their exceedingly strong antibacterial activity in both solution and components as well as their extraordinarily huge surface area. When AgNPs are applied to a wound, they adhere to the cell membrane and also enter the bacterium. Sulfur-containing proteins are present in the bacterial membrane, and the AgNPs in the cell interact with both these proteins and phosphorus-containing materials, like DNA. The DNA is shielded from the silver ions when AgNPs enter the bacterial cell because they create a low molecular weight zone in the middle of the bacterium [12]. 

Curcumin (CUR) is a natural polyphenol derived from turmeric, is a recognized agent for promoting wound healing and is acknowledged for its confirmed antioxidant, antimicrobial, and anti-inflammatory properties. Additionally, beyond its wound healing capabilities, CUR has been utilized as a reducing agent in the creation of silver nanoparticles [13]. To produce AgNPs from CUR, various chemical agents, like dimethyl sulfoxide and sodium carbonate, have been employed. However, these chemical agents can impose considerable cytotoxic effects. The selection of a suitable solvent medium and non-toxic stabilizer represents crucial considerations in the nanoparticle production [14,15].

The research combines various materials and compounds for potential therapeutic applications. Combining curcumin with silver nanoparticles and incorporating them into hydrogels made from sodium alginate and acacia gum is a strategy to potentially harness the wound healing and antimicrobial properties of each component. Curcumin is a compound found in turmeric and has known anti-inflammatory and antioxidant properties. It has been studied for its potential in promoting wound healing by reducing inflammation and supporting tissue regeneration. Silver nanoparticles are known for their antimicrobial properties. They can help prevent infection in wounds by inhibiting the growth of various microorganisms, including bacteria. Sodium alginate and acacia gum are biocompatible polymers that can form hydrogels. These hydrogels can create a moist wound environment, which is conducive to wound healing by promoting cell migration, proliferation, and tissue repair. Curcumin–silver nanoparticle-incorporated sodium alginate-co-acacia gum film hydrogels have the potential to aid in wound healing and combat wound infections due to the combined properties of their components. However, their clinical use should be based on rigorous research and assessment of their safety and efficacy. 

The novelty of this manuscript lies in its holistic approach to wound healing, incorporating multiple innovative elements, such as the use of curcumin, eco-friendly silver nanoparticle synthesis, hydrogel dressing, broad-spectrum antimicrobial action, and exceptional biocompatibility. These aspects collectively make it a promising contribution to the field of wound care. The advantages of the new hydrogel is the demonstrated effectiveness of the hydrogel dressing in combating both Gram-negative and Gram-positive bacteria. This is particularly significant in the context of rising antibiotic-resistant bacterial strains, as it offers a potential alternative for infection control in wound care. The Alg-co-AG-AgNPs hydrogel dressing exhibited faster wound healing rates compared to the control hydrogel sample. This finding suggests that the dressing may promote more rapid recovery, which can be especially beneficial in clinical settings where timely wound closure is essential. The present study specifics the synthesis of silver nanoparticles (AgNPs) through an environmentally friendly approach utilizing an aqueous solution containing hydroxypropyl-β-cyclodextrin and curcumin (βCDn-CUR). Both curcumin and hydrogel have the capacity to enhance wound healing while minimizing the formation of scars. The created wound dressing using AgNPs-SAGH holds promise as a future approach to enhance antibacterial effectiveness and support tissue recovery for skin wounds. 

## 2. Results and Discussion

### 2.1. Characterization of AgNPs

#### 2.1.1. TEM

The size and structure of the developed AgNPs using βCDn-CUR were examined by using the TEM images presented in Figure 1A,B. The analysis revealed that the nanoparticles predominantly exhibited a spherical morphology. The size range of the AgNPs ranges between 20 and 70 nm (80%) Figure 1B, and their average diameter measured 40.71 ± 18 nm (Figure 1A,B). These findings are consistent with previous literature that has reported curcumin’s capacity to act as both a reducing and capping agent [16].

#### 2.1.2. Dynamic Light Scattering (DLS)

Analysis revealed nanoparticles displaying a hydrodynamic diameter spanning 180.10 ± 8.83 nm (Figure 1C), along with a polydispersity index (PDI) of 0.195 ± 0.009. These findings suggest the potential occurrence of sequential processes involving nucleation for new nanoparticle formation and subsequent aggregation. These results align with the work of Sathishkumar et al. [17]. The low PDI value indicates that the colloidal AgNPs exhibited relatively minimal dispersion in size variability.

#### 2.1.3. Zeta Potential Measurement

The zeta potential measurement corresponds directly to the stability of the nanoparticle dispersion, as stated in reference [18]. The examination of the zeta potential indicated a negative charge present on the produced nanoparticles, quantified at approximately −20.1 ± 0.702 mV. These results closely align with values previously documented for curcumin-bio-reduced AgNPs [19].

### 2.2. Characterization of the Prepared Hydrogel Films

#### 2.2.1. Thickness

The measured thickness of the prepared hydrogel was illustrated in Table 1. The control sample (1) has the minimum thickness (0.079 mm) while AgNPs hydrogel Sample (2) has a higher thickness (0.14 mm). The presence of AgNPs in the hydrogel film caused an significant increase in thickness. This result matches the results presented in [19]. Thickness also affects other parameters, such as mechanical and barrier properties, as well as the transparency and visual appearance of the films. In order to acquire the best qualities for their intended use, biopolymer-based edible film thickness is a crucial component that needs to be carefully regulated throughout the manufacturing of the films. Figure 2 shows a visual assessment of both samples. 

#### 2.2.2. Mechanical Properties

Tensile strength (TS) and elongation at break (EAB) parameters were measured to evaluate the mechanical properties of the two prepared HG films. TS showed a significant decrease (8.48–4.27 Mpa) with the addition of AgNps (Table 1). Jaiswal et al. in 2019 [20] showed similar results, where TS of carrageenan-based films decreased with the addition of sulfur nanoparticles. The results of the EAB of the analyzed for the two prepared film samples are illustrated in Table 1. EAB significantly increased from 11.63 to 19.28% with the addition of AgNPs. The increase in EAB of the hydrogel-based films could be due to the addition of the AgNPs, as the nanoparticles act as a plasticizer and make films more flexible and less brittle. The results of the present study are in line with Oun (2017) [21], who reported an increase in the EAB with the addition of zinc and copper nanoliposomes in the carrageenan hydrogel films.

#### 2.2.3. Moisture Content

The moisture content should not exceed a certain percentage to prevent microbial growth and to keep the structural integrity of the hydrogel film. In the current study, a slight decrease from 18.48% to 16.33% in moisture content was observed with the addition of AgNPs. The noticed slight decrease in the moisture content of the films when adding the AgNPs could be due to the hydrophobic nature of these nanoparticles. Koneru (2020) [22] reported a decrease in the moisture content of hydrogel films, based on cellulose, when incorporated with nanoparticles consisting of carboxymethylcellulose–grapefruit seed extract nanoparticles.

#### 2.2.4. Transparency of the Films

The synthesized hydrogel films loaded with AgNPs have been examined for transparency and color parameters, including Lightness (L), a*, b*, and ΔE*. The addition of AgNPs had a significant impact on the transparency of the films (Table 2). 

With AgNPs added, the transparency dropped from 79 to 21%. The outcomes of the present study are consistent with those of a prior investigation, which found that the addition of oregano and black cumin essential oils reduced the transparency of starch-based films [22].

The synthesized nano-silver-loaded hydrogel films showed a slight decrease in Lightness (L), from 90.32 to 87.4%, with the addition of AgNPs. The a* value of the films varied from 0.03 to 0.22, whereases the b* value ranged from 0.9 to 3.42. As mentioned in Table 2, the films showed (b*) yellowness in the presence of the AgNPs. The significant variation of ΔE values (2.67–4.92) confirms the overall color changes made by the addition of AgNPs to the films.

#### 2.2.5. Scanning Electron Microscopy

Figure 3 displays the SEM outcomes of the ALg-AG film samples with the additional AgNPs. In contrast to the films with AgNPs, the control film (1) with Alg and AG displayed a structure with some pores on the film surface. The protrusion is visible in the cross-sectional photo of the control sample as well. The aggregation that resulted from the uneven distribution of hydrophobic components during the film-forming technique may have contributed to the roughness of the film sample (2). Additionally, the AgNP-incorporated film samples had uniform structures, smooth surfaces with fewer particles, and no holes or fractures. Similar findings were reported by Oun, (2017) [23], in which the AgNPs were evenly dispersed throughout the hydrogel films’ polymer matrix. 

### 2.3. In Vitro Cytocompatibility and Hemocompatibility

The literature extensively acknowledges the biocompatible characteristics of Alg–AG film hydrogels, as highlighted in Gupta et al., 2018, Pertile et al., 2012 [24,25]. The biocompatibility of hydrogels containing AgNP-incorporated Alg–AG was assessed using three distinct mammalian cell lines. The evaluation of cytotoxicity through the MTT assay demonstrated that AgNP-incorporated ALg–AG maintains cytocompatibility, with all tested cell lines exhibiting favorable survival rates (Figure 4a). Moreover, we conducted a comparative assessment of the biocompatibility between the control hydrogel-free (1) and the test (2) AgNPs encapsulated within Alg–AG using MSTO, U251, and Panc1 cell lines. The outcomes revealed that the control exhibited cytotoxic properties across all examined cell lines, leading to reduced cell viability in contrast to AgNPs integrated into ALg–AG (significance level of *p* < 0.001), as illustrated in Figure 4b. These findings imply that ALg–AG effectively regulates the release of AgNPs, thereby mitigating the cytotoxic impact on mammalian cells. This evidence lends support to the potential utility of AgNPs-incorporated as hydrogel dressings for wound management.

Alg–AG has been acknowledged for its hemocompatible attributes, a feature that has led to its inclusion in exclusive wound dressing products, as documented in [26]. In this present investigation, AgNPs were synthesized using deionized water, prompting the hypothesis that AgNP-incorporated Alg–AG hydrogels could possess hemolytic characteristics. The test outcomes revealed that AgNP-loaded Alg–AG hydrogels displayed a hemolysis percentage of 7.05 ± 1.12%. The increased hemolysis percentage observed in the tested hydrogels could be attributed to the utilization of deionized water as an isotonic solution during the AgNPs synthesis process. In the case of chronic wounds, necrotic tissue or slough might be present at the wound bed, which could potentially mitigate the hemolytic response of these hydrogels. Future investigations focusing on the synthesis of AgNPs using βCDn–CUR dissolved in an isotonic solution may offer enhancements in the hemocompatibility of these hydrogels.

### 2.4. Transparency Test

The progression of wound healing holds significant clinical importance [27]. Typically, this process necessitates the removal of a dressing, a procedure that could disrupt the granulation tissue and potentially inflict trauma upon the wound. The inclusion of a dressing with the capability for noninvasive monitoring could prove advantageous for facilitating wound healing. The investigation conducted here, which was specifically focused on the transparency feature of the assessment of AgNP-loaded Alg–AG, was performed by reading text of various colors on a white laminated paper film through the experimental hydrogels. 

### 2.5. Investigation of Antimicrobial Properties

The antimicrobial properties of silver nanoparticles have been extensively investigated. AgNPs have the capability to enhance the permeability of the cell membrane, disrupt DNA replication, denature bacterial proteins, and release silver ions within the bacterial cell. In the current study, hydrogels containing Sodium Alginate–Gum loaded with colloidal silver nanoparticles (AgNPs) were subjected to testing against *S. aureus* and *E. coli* using the disc diffusion assay after 24 h. The free hydrogel (1) did not exhibit any antimicrobial activity. In contrast, hydrogel loaded with AgNPs (2) exhibited substantial antimicrobial activity (with a statistical significance of *p* < 0.001) against both tested microbial strains, as shown in Figure 5. These findings validate the extensive range of antimicrobial effects exhibited by an Alg–AG film infused with AgNPs. Furthermore, the enhanced antimicrobial potency of an AgNP-impregnated Alg–AG film is evident (as shown in Figure 5) in its ability to combat *E. coli* more effectively than *S. aureus* (with a significance level of *p* < 0.001). This variance in antimicrobial performance can be attributed to the variations in the cellular structures of Gram-positive and Gram-negative bacteria. The capabilities of AgNPs to induce a separation between the cytoplasm and the bacterial cell wall has been documented as a mechanism resulting in the death of *E. coli* Conversely, in the case of *S. aureus*, AgNPs exhibit an alternative mode of action by impeding the synthesis of the bacterial cell wall, ultimately leading to bacterial cell death [15].

Translating curcumin–silver nanoparticle-incorporated sodium alginate-co-acacia gum film hydrogels from a research concept to clinical practice involves a multifaceted approach. It encompasses clinical validation, regulatory approvals, production scalability, quality control, cost-effectiveness, healthcare professional training, and patient acceptance. Successfully navigating these aspects is crucial for the adoption and integration of this innovative wound dressing technology into routine clinical care.

## 3. Conclusions

The present study demonstrates the creation of AgNP-incorporated Alg-AG film hydrogels, encompassing meticulous physicochemical and in vitro assessments. This approach enhances effectiveness and reduces the risk of untimely structural issues in designed biomaterials both prior to and following specific applications. Silver nanoparticles (AgNPs) were synthesized using an eco-friendly approach, employing curcumin. TEM, DLS, and zeta potential have been used for the characterization of the synthesized silver nanoparticles. The findings underscore the successful synthesis of AgNPs utilizing the green chemistry principle via βCDn–CUR, with their subsequent integration into Alg-AG to yield hydrogels primed for potential wound dressing use. These hydrogels exhibit wide-ranging antimicrobial effects. Additionally, they showcase compatibility with the assessed cell lines, emphasizing their value. The considerable moisture content and commendable transparency the management of persistent wounds characterized by substantial microbial presence.

## 4. Materials and Methods

### 4.1. Materials

Sodium alginate (Alg) and gum arabic (Ga) were purchased from Sigma-Aldrich (St. Louis, MO, USA). Methylene bisacryl-amide (MBA) (Fluka, Buchs, Germany) and potassium persulfate (KPS) (Merck, Darmstadt, Germany) were used as the crosslinker and initiator, respectively. 

#### 4.1.1. Tissue Culture and Silver Nitrate

Three types of tissue cultures (MSTO, U251MG (U251), and Panc1 cell lines) were procured from ATCC (Teddington, UK). Defibrinated whole blood from horses was acquired from TCS Biosciences Ltd., Buckingham, UK.

Silver nitrate (AgNO3, with a purity of 99.9%), β-cyclodextrin (β-CDn, with a purity of 99%), and curcumin (Cur, with a purity of 98%) (El Nasr Pharmaceutical Chemicals Co., Cairo, Egypt). 3-(4.5-dimethylthiazol-2-yl)-2.5-diphenyl tetrazolium bromide (MTT) was purchased by Sigma-Aldrich (St. Louis, MO, USA).

#### 4.1.2. Bacterial Tested Strains

Gram-negative bacteria *E. coli* (number: 25,922) and Gram-positive bacteria *S. aureus* (number: 25,923) were supplied from the Bacteriology Unit in National Research Centre, Egypt (NRC). Both microorganisms were preserved in a freeze-dried state at −20 °C. Initial cultures of both S. aureus and *E. coli* were reactivated by applying them onto sterile tryptone soy agar (TSA) obtained from Sigma-Aldrich, UK. This agar was prepared following the provided instructions and sterilized via autoclaving before being utilized. Subsequently, the cultures were incubated at a temperature of 37 °C. Overnight broth cultures were then accurately prepared using the initial stock plates. 

### 4.2. Preparation of βCDn–CUR Complex

The complex was synthesized using the solvent evaporation technique [17]. In a concise manner, a solution of CUR (0.70 g/38 mL acetone) was gradually introduced into an aqueous solution of βCDn (4.0 g/13 mL deionized water) with stirring at room temperature to facilitate the gradual and complete removal of acetone through evaporation. Subsequently, the mixture underwent centrifugation, and the resulting aqueous supernatant containing the βCDn–CUR complex was subjected to filtration and lyophilization after being frozen [28].

### 4.3. Synthesis and Characterization of AgNPs

The creation of AgNPs using βCDn–CUR as an environmentally eco-friendly method through the reduction of silver nitrate (AgNO_3_) through utilizing an aqueous (0.20 g) βCDn–CUR solution, a solution was prepared by dissolving it in deionized water (19 mL). This βCDn–CUR aqueous solution was introduced drop by drop with continuous stirring into a 1 mM AgNO_3_ aqueous solution (45 mL) under boiling conditions within conical flasks. The combined solutions underwent boiling for a duration of 3 h to affect the reduction of Ag ions, followed by a 30 min cooling period at room temperature. To ensure a light-free environment and prevent any photochemical reactions, the flask was covered with aluminum foil throughout the reduction process.

The morphology of AgNPs was observed through the use of a transmission electron microscope (TEM, JEM-2010 HR, Tokyo, Japan). A droplet of aqueous colloidal AgNPs was deposited onto a carbon-coated 300 mesh copper grid (provided by Agar Scientific, Redding, CA, USA), allowed to stand for 30 min, washed, and then air-dried within a covered container at room temperature. TEM imaging was conducted with an electron microscope operating at 80 keV. A range of magnifications was used for capturing images. To determine size distribution, approximately 100 AgNPs were selected randomly and measured using ImageJ software. The identical instrument was employed to acquire the DLS. Five successive measurements were carried out at a temperature of 25 °C, with samples being allowed to equilibrate for a period of 2 min before the measurements commenced. The resulting data were averaged to determine the mean size. The Malvern Zeta/sizer Nano-ZS instrument (Zetasizer Nano ZS90; from Malvern, UK) at the National Research Center, Egypt (NRC) was utilized to measure the zeta potential and hydrodynamic diameter. Five consecutive measurements were taken and then averaged to discover the zeta potential.

#### Synthesis of Sodium Alginate-Co-Acacia Gum-Loaded AgNP Hydrogel Film

AgNPs (1 mg/mL) were added to the aqueous solution of sodium alginate (1% *w*/*v*) in the ratio of 2:3 (Polymer solution I). Hydrogels were prepared by the dropwise addition of aqueous solution of acacia gum (AG) (0.1% *w*/*v*) into polymer solution I in a ratio of 1:2 (Polymer solution II). Crosslinker methylene bisacrylamide (MBA) (1% of Polymer solution II) was added dropwise under constant stirring. The obtained solution was poured onto a Petri plate and left to dry for 48 h at room temperature. After drying, the film was evaluated visually and subjected to further examination. The control hydrogel sample was prepared similarly but without the addition of AgNPs in Polymer solution I [28].

### 4.4. Characterization of the Prepared Hydrogel Films

#### 4.4.1. Thickness

The thickness of the prepared hydrogel film samples can vary depending on the type of material and the process used for the preparation. To determine the thickness of the films produced, a digital micrometer (Guilin Millimeter Industry Co., Ltd., Guilin, China) was utilized. The thickness measurements were taken in a different position of the film, and the average value was calculated. 

#### 4.4.2. Mechanical Properties

By altering the composition of the film or the production parameters, the mechanical characteristics of the edible film may be changed. The kind and proportion of the polymer, plasticizer, and other additives, as well as how they interact with one another, can all have an impact on the tensile strength. Using a texture analyzer (XT plus, Stable Micro Systems, Godalming, England), we measured the mechanical characteristics of the hydrogel films, especially their tensile strength (TS) and percentage elongation at break (EAB), in accordance with the recommended ASTM D882 technique. Film strips that were 60 mm long and 7 mm broad were utilized for the test. The values of the TS and EAB for the film samples were calculated using the formulae listed below.

(1) $$TS=\frac{F}{A}$$

*F* is the maximum force, *A* is the cross sectional area of the film.

(2) $$EAB\;\left(\%\right)=\frac{L_{f}-L_{i}}{L_{i}}$$

*L_f_* is the final length of the film.

*L_i_* is the initial length of the film.

#### 4.4.3. Moisture Content

It is crucial to consider the hydrogel films’ moisture content since it might impact the food’s quality, safety, and shelf life. We measured the moisture content (MC) of the hydrogel film strips, which measure 1 cm by 3 cm. Equation (3) was used to compute the weight difference between the film strips before (*W*_1_) and after (*W*_2_) drying, which took place at 105 °C.

(3) $$MC=\frac{W_{1}-W_{2}}{W_{1}}$$

#### 4.4.4. Transparency of the Films

Transparency and color parameters are important factors as they affect the visual appearance, freshness, and quality parameters of food products. The transparency of the prepared hydrogel film samples was measured at a wavelength of 550 nm by using a spectrophotometer (ONDA-Vis spectrophotometer, V-10 Plus, ONDA, Padova, Italy) according to the method described by Bhatia (2023). The surface color analysis of the Alg–AG-based films was carried out by using a colorimeter (Konica Minolta, Tokyo, Japan), and represented as L* (lightness), a* (red/green), and b* (yellow/blue). The film samples were placed on the surface of a standard plate (L* = 100), and the color parameters L*, a*, and b* were calculated. Equation (4) was used to calculate the ΔE (the overall color difference).

ΔE* = {(ΔL*)^2^ + (Δa*)^2^ + (Δb*)^2^}^1/2^ (4)

#### 4.4.5. Scanning Electron Microscope (SEM)

JEOL SEM 6000 Neo scope desktop SEM image scanning microscopes are used to characterize morphology. Fractions were frozen in liquid nitrogen to create fiber cross-sections. Samples were coated with a thin coating of gold using a gold-sputter in preparation for SEM inspection. EDS has assessed the elemental analyses of the manufactured PVDF hollow fibers.

### 4.5. In Vitro Cytocompatibility Study

To examine the cytocompatibility of sodium alginate gum hydrogel incorporated with AgNPs, an in vitro cell viability assessment was carried out utilizing three distinct human cancer cell lines originating from various tissues were used, namely U251MG (human glioblastoma), MSTO (human mesothelioma), and Panc1 (human pancreatic ductal adenocarcinoma), and all the cell lines were cultivated in Dulbecco’s Modified Eagle’s Medium (DMEM) supplemented with fetal bovine serum (FBS) and antibiotic antimycotic. The cultures were maintained at 37 °C in a humidity-controlled incubator with 5% CO_2_.

Hydrogel films (control) or with AgNPs (test) were subjected to agitated conditions (160 rpm) at 4 °C. Subsequently, these samples (both control and test) were sectioned into 10 mm discs, adhering to aseptic practices, and the temperature was adjusted to 37 °C prior to use. For experimentation, 30,000 cells were seeded per well in a 24/well plate and cultured for 24 h at 37 °C within a 5% CO_2_ incubator. Subsequently, the test cells were subjected to exposure either to hydrogel or AgNP-incorporated hydrogel (8 mm discs) for 24 h to assess their impact on cell viability. The standard MTT cytotoxicity assay, a 5 mg/mL MTT solution (from Sigma, Gillingham, UK), was introduced into all the wells. Subsequently, the cells were incubated for a duration of 2 h. Following this, the formazan crystals were dissolved using dimethyl sulfoxide (DMSO) in combination with Sorensen’s glycine buffer (pH 10.5). Cell viability was determined by calculating the average absorbance measured at 540 nm. The outcomes were subjected to statistical analysis using a two-way analysis of variance (ANOVA) coupled with a Tukey’s multi-comparisons test using GraphPad Prism.

### 4.6. AgNP-Loaded Sodium Alginate-Co-Acacia Gum Hydrogel Hemocompatibility Determination

Defibrinated horse whole blood was subjected to two washes using commercially available normal saline at a pH of 5.5. Following this, the blood cells were resuspended in normal saline. Discs of AgNPs-loaded Hydrogel films measuring 8 mm in diameter were prepared by utilizing a biopsy punch and subsequently placed in test Eppendorf tubes. Each of these tubes contained 1.9 mL of horse blood cells suspended in normal saline. For the positive control (+ve), blood cells were suspended in distilled water, while for the negative control (−ve), blood cells were suspended in normal saline. All the Eppendorf tubes, both test and control, were placed in incubation at 4 °C for a period of 2 h, with periodic inversion every 15 min. Upon completion of the incubation, the Hydrogel discs 8 mm were removed from the test Eppendorf tubes. Subsequently, all the tubes were subjected to centrifugation at 3000 rpm for 10 min at a temperature of 4 °C. Following centrifugation, the supernatant was decanted, and absorbance was measured at 540 nm to determine the percentage of hemolysis (% Hemolysis).

(5) $$Hemolysis\;\left(\%\right)=\frac{\left(Sample\;Absorbance\right)\left(Absorbance\;of\;-ve\;control\right)*100}{\left(Absorbance\;of\;+ve\;control\right)\;\left(Absorbance\;of\;-ve\;control\right)}$$

### 4.7. Disc Diffusion Assay

The bactericidal activity of AgNP-loaded sodium alginate hydrogel was examined against Gram-negative *E. coli* and Gram-positive *S. aureus* bacteria by employing the disc diffusion assay. Controls consisted of sodium alginate–gum hydrogel films and the test contain hydrogel films loaded with βCDn. Discs measuring 8 mm in diameter were aseptically positioned on TSA plates that had been previously spread with an overnight culture of either *E. coli* or *S. aureus*. Subsequent to incubation at 37 °C for a duration of 24 h, the zones of inhibition were measured. The statistical analysis involved presenting the data as mean ± standard deviation (SD) and conducting a two-way analysis of variance (ANOVA) alongside a Tukey’s multi-comparisons test. Antioxidant analysis was performed using DPPH Assay. The potential antioxidant properties of AgNPs, synthesized via βCDn-CUR, were assessed by employing the 2,2-diphenyl-1-picrylhydrazyl (DPPH) radical scavenging assay. For this assay, a mixture consisting of 1 mL of methanolic DPPH solution (80 μg/mL) and 1 mL of the test colloidal AgNPs were combined and incubated for 30 min in a dark environment at room temperature. Subsequently, the absorbance was measured at 517 nm, and the percentage of antioxidant effect (%AE) was calculated as an indicator of the free radical scavenging potential.

(6) $$Antioxidant\;effect\;\left(\%\;AE\right)=\frac{Control\;Absorbance-Sample\;Absorbance}{Control\;Absorbance\times 100}$$

Observing the progression of healing without having to remove the dressing could significantly reduce disruption to the granulating tissue. With the objective of utilizing the hydrogel for wound dressing purposes, the transparency of AgNP-incorporated sodium alginate-co-acacia gum hydrogels was evaluated through a simulated test. Both hydrogels and AgNP-loaded hydrogels were placed onto a laminated film of paper containing text of various colors. The clarity of the text beneath the hydrogel was examined to ascertain whether the healing tissue at the wound site could be observed through these hydrogels.

## Figures and Tables

**Figure 1:** (**A**) TEM characterization of AgNPs, (**B**) size distribution as measured by TEM analysis and calculated with 100 nanoparticles, and (**C**) DLS data of AgNPs with size distribution.

**Figure 2:** A photo for the two prepared HG film: (**1**) the control film hydrogel, (**2**) HG film loaded with AgNPs.

**Figure 3:** SEM of the prepared HG Film: (**1**) control; (**2**) film loaded with AgNPs.

**Figure 4:** Cytocompatibility test results. (**a**) Bar graph showing the cell viability (%) after 24 h exposure to control hydrogel (1) and AgNP-loaded hydrogel (2). (**b**) Hydrogel-free (1) and the test (2) AgNPs encapsulated within Alg–AG using MSTO, U251, and Panc1 cell lines.

**Figure 5:** Antimicrobial disc diffusion assay results for free hydrogel and AgNP-incorporated hydrogel against *E. coli* and S. *aureus* at 24 h. (n = 10; error bars = SD).

**Table 1:** The thickness, tensile strength, elongation at break, moisture content of both samples.

Film Sample	Thickness (mm)	TS (Mpa)	EAB (%)	Moisture Content (%)
1	0.079	8.48	11.63	18.48
2	0.14	4.27	19.28	16.33

**Table 2:** Transparency and color parameters of the prepared hydrogel films.

HG Sample	Transparency (%)	L	a*	b*	ΔE*
1	73.81	90.32	0.03	0.90	2.67
2	61.43	87.40	0.22	3.42	4.92

L: lightness; a*: green-red color; b*: blue-yellow color; ΔE*: overall color variation.

## Data Availability

The data presented in this study are available upon request from the corresponding author.
